# Evaluation of the Antimalarial Activity of the Leaf Latex of *Aloe weloensis* (Aloaceae) against *Plasmodium* Parasites

**DOI:** 10.1155/2021/6664711

**Published:** 2021-06-16

**Authors:** Gedefaw Getnet Amare, Amsalu Degu, Peter Njogu, Zemene Demelash Kifle

**Affiliations:** ^1^Department of Pharmacy, College of Medicine and Health Sciences, Wollo University, Dessie, Ethiopia; ^2^Department of Pharmaceutics and Pharmacy Practice, School of Pharmacy and Health Sciences, United States International University-Africa, Nairobi, Kenya; ^3^Department of Pharmaceutical Chemistry, School of Pharmacy, University of Nairobi, Nairobi, Kenya; ^4^Department of Pharmacology, School of Pharmacy, College of Medicine and Health Sciences, University of Gondar, Gondar, Ethiopia

## Abstract

**Background:**

The lack of available vaccines and the emerging resistance to antimalarial drugs have provided the necessity to find noble antimalarial plant-based medicines. The leaf latex *Aloe weloensis* has been used in folk medicine against malarial and other human ailments in Ethiopia. Hence, the present study aimed to investigate the antimalarial activity of the leaf latex of *A. weloensis* against *Plasmodium* parasites.

**Materials and Methods:**

The prophylactic and curative models were employed to determine the in vivo antimalarial activity of the leaf latex *A. weloensis* against *P. berghei* infected mice, and the antioxidant activity of the latex was assessed using diphenyl-1-picrylhydrazine (DPPH) assay. Female mice were recruited for toxicity study, and the leaf latex was administered to fasted mice at a dose of 5000 mg/kg. The mice were kept under continuous observation for fourteen days for any signs of overt toxicity.

**Results:**

The leaf latex of *A. weloensis* was safe up to 5000 mg/kg, and the latex endowed free radical inhibition activity (IC_50_ = 10.25 *μ*g/ml). The latex of *A. weloensis* leaf demonstrated the inhibitory activity against the 3D7 strain of *P. falciparum* (IC_50_ = 9.14 *μ*g/ml). The prophylactic and curative effect of the latex was found to be dose-dependent. The mice's parasitemia level was significantly (*p* < 0.001) reduced at all tested doses of the leaf latex compared to negative control in the curative test. Parasitemia reduction was significant (200 mg/kg, *p* < 0.01, and 400 and 600 mg/kg, *p* < 0.001) in the prophylactic test compared to the control. In addition, the leaf latex significantly (*p* < 0.01) improved mean survival time, packed cell volume, rectal temperature, and bodyweight of *P. berghei* infected mice.

**Conclusion:**

The leaf latex of *Aloe weloensis* was endowed with the antimalarial activity at various doses, corroborating the plant's claimed traditional use.

## 1. Background

Plants and plant extracts possess a wide margin of safety and show potential effectiveness in treating various diseases [1, 2]. Medicinal plants are the primary resource for treating malaria infections in Africa since healthcare facilities are limited [3]. The currently available antimalarial drugs such as quinine, halofantrine, mefloquine, chloroquine, and artemisinin are of plant origin [4–6].

The lack of available vaccines and the emerging resistance to antimalarial drugs have provided the necessity to find noble plant-based antimalarial drugs [7–9]. Developing noble antimalarial agents is imperative to overcome the challenges posed by the development of antimalarial drug resistance. Nature has gifted various plants with a potential effect against *Plasmodium* parasites [10–12].

Aloe species have been used as topical and oral therapeutic agents due to their health, beauty, medicinal, and skincare properties. They have demonstrated antibacterial, antitumor, anti-inflammatory, antiarthritic, antirheumatoid, anticancer, and antidiabetic activities [13]. The latex of *Aloe weloensis* leaf showed an antibacterial effect against Gram-negative and Gram-positive strains [14]. The plant's leaf latex has been used in folk medicine against malarial and other human ailments in Ethiopia [15]. Previously, the leaf latex *Aloe weloensis* showed a significant antimalarial effect in Peter's (4-day suppressive) test and safe at 2000 mg/kg [16]. Besides, phytochemical studies showed that this plant's leaf latex was endowed with flavonoids, glycosides, anthraquinones, saponins, terpenoids, and tannins with prominent antimalarial activities in various plant extracts [12, 17–19]. Eventhough few investigations have been conducted previously, there was a paucity of comprehensive studies in other models (prophylactic and curative models) and in vitro studies (DPPH assay). Therefore, this study was aimed to investigate the antimalarial activity of the leaf latex of *A. weloensis* against *Plasmodium* parasites using prophylactic and curative models.

## 2. Materials and Methods

### 2.1. Collection and Preparation of Leaf Latex of *Aloe weloensis*

The leaf of *A. weloensis* was collected for identification from northeast Ethiopia (Guba Lafto) in May 2020. The plant was identified by Ms. Habtam G (botanist) with voucher specimen number HG010/20. After identification, the leaf *A. weloensis* was cut near the stem and inclined towards the collecting plate to gain the latex. The latex was dried under shade at room temperature with optimal ventilation. The dried latex was kept in a clean vial and stored in a dessicator until used for the experiment.

### 2.2. Experimental Animals and Parasites

Healthy Swiss albino mice of either sex weighing 20–35 grams and aged 2-3 months were used in the study. The mice were obtained from Wollo University, Department of Pharmacology. The mice were kept in plastic cages at room temperature and 12 h light and 12 h dark cycle, with free access to pellet food and water in the laboratory [17, 18]. The mice were acclimatized to laboratory condition for one week before the initiation of the experiment. The *P. berghei* ANKA strain was obtained from Ethiopian Public Health Institute, while the 3D7 strain of *P. falciparum* was obtained from Italy. The *P. berghei* parasite was maintained by serial blood passage from infected mice to uninfected ones on a seven-day basis. This study was carried out based on the guide for the care and use of laboratory animals [17, 20, 21].

### 2.3. Acute Oral Toxicity Study

An acute oral toxicity study was carried out based on the Organisation for Economic Co-operation and Development (OECD) guidelines 425 [22]. Female mice were recruited for the toxicity study since they are more sensitive than male mice. One female Swiss albino mouse fasted for 4 h, and the animal's fasting bodyweight was measured [17]. Then, the leaf latex was administered to the mouse at a dose of 5000 mg/kg. The mouse was then kept under strict observation of physical and behavioral changes for one day, with special attention during the first 4 h. Following the result from the first mouse, another four mice fasted for 4 h, and then, the latex was administered to each mouse at the dose of 5000 mg/kg and was observed in the same manner. The observation was continued for fourteen days for any signs of overt toxicity.

### 2.4. In Vitro Antioxidant Activity of the Leaf Latex *Aloe weloensis*

Antioxidant activity of the latex of *A. weloensis* leaf was evaluated using DPPH-free radical scavenging assay following the method of MacDonald-Wicks et al. [23] as previously described by Sanchez-Moreno et al. [24]. A 3 ml of 0.1 mM DPPH in methanol was mixed in 1 ml methanolic solution of different concentrations (12.5–400 *μ*g/ml) of the latex and incubated in the dark for 30 min at room temperature. Ascorbic acid was used as a standard antioxidant. After 30 min, the absorbance of the mixture and the control at 517 nm was read by using a UV spectrophotometer. The test was conducted in triplicate, and the percent of scavenging of inhibition was calculated as follows:

(1) $$\begin{array}{c} \%\text{of free radical scavenging}=\frac{\left(\text{absorbance of control}-\text{absorbance of sample}\right)}{\text{absorbance of control}}\times 100. \end{array}$$

### 2.5. In Vitro Antimalarial Evaluation of the Leaf Latex of *Aloe weloensis*

Chloroquine-sensitive 3D7 strain of *P. falciparum* was used to determine the in vitro antimalarial activity of the leaf latex of *A. weloensis*. *Plasmodium falciparum* culture was maintained following previously described methods with some modifications [19, 25]. *Plasmodium falciparum* (suspension of 3D7) synchronized in 5% sorbitol to ring stage was seeded (200 *μ*l/well with 2% ring stages and O^Rh+^red blood cells at 2% hematocrit) in 96-well tissue culture plates. The latex of *A. weloensis* leaves in different concentrations (10–320 *μ*g/ml) was added to these wells. The same chloroquine concentration was used as the standard control, and dimethyl sulfoxide was used as the negative control. The parasites were cultured for 30 h in the desiccator and then incubated (37°C) for 72 h in 2% O_2_, 5% CO_2,_ and 93% N_2_ [18, 19]. The infected red blood cells (RBCs) were transferred into a freshly prepared complete medium to propagate the culture. After 72 h incubation, the cultures were preserved (−20°C), and the parasites were harvested. The thin blood smears were prepared and fixed with methanol and stained with 10% Giemsa for 30 min to evaluate the parasites' growth stage. The parasitemia was examined under the microscope, and IC_50_ was determined by plotting the latex concentration on the percentage of growth inhibition. Percentage growth inhibition of the parasites was determined by using the following formula [18, 25].

(2) $$\begin{array}{c} \%\text{ of growth inhibition}=\frac{\left(\text{mean parasitemia of control}-\text{mean parasitemia of the sample}\right)\times 100}{\left(\text{mean parasitemia of control}\right)}. \end{array}$$

### 2.6. Parasites Inoculation

*Plasmodium berghei* ANKA strain was used for induction of malaria in experimental mice. The parasites were maintained by intraperitoneal serial passage of blood, and the parasitemia level (30–37%) of *P. berghei* infected donor mice was determined [26, 27]. The donor mouse was anaesthetized by pentobarbitone at 150 mg/kg intraperitoneally (i.p.). Then, infected blood was collected by cardiac puncture into a heparinized vacutainer tube containing trisodium citrate (0.5%). The blood was then diluted in normal saline (0.9%), so that the final suspension would have about 1 × 10^7^ parasitized red blood cells (PRBCs) in 0.2 ml suspension [17, 18]. Each mouse was infected intraperitoneally with 0.2 ml of 1 × 10^7^*P. berghei* parasitized RBCs.

### 2.7. Dosing and Grouping of the Animals

The mice were randomly divided into five groups (*n* = 6). Group I (negative control) was treated with 10 mg/kg 2% Tween-80 in distilled water (TW80). Groups II, III, and IV were treated with 200, 400, and 600 mg/kg doses of the leaf latex, respectively. Group V was treated with the standard drug, chloroquine (25 mg/kg) [17, 20]. Effective dose selection was calculated as per the oral acute toxicity test of the Organisation for Economic Co-operation and Development guidelines and pilot experiments. Since there were no observed signs of toxicity at 2000 mg/kg, 1/20^th^ (100 mg/kg), 1/10^th^ (200 mg/kg), and 1/5^th^ (400 mg) of 2000 mg/kg doses were considered for the pilot test. After the pilot experiment, we increased the doses until we get an effective dose. Accordingly, 200, 400, and 600 mg/kg doses were considered effective doses to be considered in the main experiment.

### 2.8. Antimalarial Activity of the Leaf Latex of *A. weloensis* in the Curative Test (Rane's Test)

On the first day (day 0), the mice were injected intraperitoneally with a standard inoculum of 1 × 10^7^*P. berghei* infected erythrocytes. After seventy-two hours, the mice were randomly assigned into five groups (*n* = 6). Group I was treated with vehicle; groups II, III, and IV were treated three doses of the latex of *A. weloensis*, respectively. Group V was treated with chloroquine daily for five days. Thin blood films were prepared from each mouse's tail blood daily for five days to determine parasitemia levels and mean survival time for each group [17, 18, 27].

### 2.9. Antimalarial Activity of the Leaf Latex of *A. weloensis* in the Prophylactic Test

Mice were randomly assigned into five groups (*n* = 6) and treated with a single dose according to their respective grouping. Then, after 24 h (day 0), each mouse was injected intraperitoneally with 0.2 ml infected blood containing 1 × 10^7^*P. berghei* parasitized RBCs. After 72 h (day 3 postinfection), blood samples were collected from each mouse's tip tail, and slides were prepared. Then, % inhibition, parasitemia level, and survival time were determined [17].

### 2.10. Peripheral Blood Smears Preparation

Thin smears of blood were made from each mouse's tail. The smears were applied on microscopic slides, and the blood was drawn evenly across a second slide to make thin blood films and allowed to dry at room temperature. Then, they were fixed with absolute methanol and stained with 10% Giemsa stain (pH = 7.2) for 15 min.

### 2.11. Parasitemia Determination

Each stained slide for each mouse was examined under a microscope. The parasitemia level was determined by counting the number of parasitized erythrocytes in random fields of the microscope. Percent parasitemia and percent suppression were calculated by using the following formula.

(3) $$\begin{array}{c} \%\text{ of parasitemia}=\frac{\left(\text{number of parasitized RBC}\right)\times 100}{\left(\text{total number of RBC}\right)},\\ \%\text{ of suppression}=\frac{\left(\text{mean parasitemia of negative control}-\text{mean parasitemia of the treated group}\right)\times 100}{\left(\text{mean parasitemia of negative control}\right)}. \end{array}$$

### 2.12. Determination of Mean Survival Time

Mean survival time (MST) is another parameter that is commonly used to evaluate the efficacy of antimalarial plant materials. Mortality was monitored daily, and the number of the days from the time of infection up to death was recorded for each mouse in the treatment and control groups throughout the follow-up period. The MST was calculated for each group by using the following formula.

(4) $$\begin{array}{c} \text{MST}=\frac{\text{sum of survival time of all mice in a group}\left(\text{days}\right)}{\text{total number of mice in that group}}. \end{array}$$

### 2.13. Packed Cell Volume Measurement

The packed cell volume (PCV) was measured to predict the effectiveness of the test latex in preventing hemolysis from the high level of parasitemia. Blood was collected from each mouse's tail in heparinized microhematocrit capillary tubes by filling three-quarters of its volume. The tubes were sealed by sealant and placed in a microhematocrit centrifuge with the closed ends outwards.

The blood was then centrifuged at 12,000 rpm for 15 min. The tubes were then taken out of the centrifuge, and PCV was determined using a standard microhematocrit reader. The PCV of each mouse was then measured before infection and on day four after infection using the formula [17, 20, 26].

(5) $$\begin{array}{c} \text{PCV}=\frac{\left(\text{volume of erythrocytes in a given volume of blood}\right)}{\left(\text{total blood volume}\right)}. \end{array}$$

### 2.14. Determination of Bodyweight and Temperature Changes

The bodyweights of the mice were determined to observe whether the leaf latex was prevented weight loss for Peter's test. The bodyweight of each mouse was measured before infection (day 0) and on day 4 using a sensitive digital weighing balance. Rectal temperature was also measured before infection, four hours after infection, and then daily by a digital thermometer.

### 2.15. Statistical Analysis

The results of the study were expressed as the mean ± standard error of the mean. Statistical analysis of the data was carried out with a one-way analysis of variance followed by the Tukey post hoc multiple comparison test. Significant differences were set at *p* < 0.05.

## 3. Results

### 3.1. Acute Toxicity

The mice were observed for gross signs of toxicities such as loss of appetite, hair erection, lacrimation, tremors, convulsions, salivation, diarrhea, and mortality during the experiment. Nonetheless, in the acute toxicity test, no sign of toxicity or mortality was observed in mice after oral administration of the leaf latex at 5000 mg/kg doses, signifying that LD_50_ was greater than 5000 mg/kg.

### 3.2. Antioxidant Activity of the Leaf Latex of *Aloe weloensis*

The antioxidant capacity of the latex was evaluated using the DPPH-free radical assay method. Qualitative detection showed that the color of the test solution changed from violet to a slightly yellow color. The finding of the study showed that antioxidant activity (*p* < 0.001) of the latex was concentration-dependent with an IC_50_ value of 10.25 *μ*g/ml (Table 1).

### 3.3. The Effect of the Leaf Latex of *A. weloensis* on *P. falciparum* Growth in Culture

After 72 h incubation, the latex of *A. weloensis* potentially inhibited (*p* < 0.001) the growth of the 3D7 strain of *P. falciparum*. The finding showed that the latex was active against *P. falciparum* parasites, and growth inhibition was dose-dependent (Figure 1). The IC_50_ of the latex and chloroquine was 9.14 and 0.12 *μ*g/ml, respectively.

### 3.4. The Effect of the Leaf Latex of *Aloe weloensis* in the Curative Test

The finding showed that parasitemia reduction was significant (*p* < 0.001) at 200, 400, and 600 mg/kg doses of the latex with suppression of 36%, 58%, and 74%, respectively (Table 2). The result showed that all doses of the latex endowed the curative effect as compared to the control. The curative effect of 200 mg/kg dose was significantly (*p* < 0.01) lower than chloroquine (*p* < 0.001). All tested doses of the latex significantly (*p* < 0.01) improved the mean survival time of the mice compared to the negative control. Nonetheless, the survival time of the mice treated with the lowest dose (200 mg/kg) was significantly (*p* < 0.01) lower than chloroquine.

### 3.5. The Effect of *A. weloensis* Leaf Latex on PCV, Rectal Temperature, and Bodyweight

In this study, the leaf latex at 400 and 600 mg/kg doses significantly (*p* < 0.01) prevented packed cell volume and reduced rectal temperature of *P. berghei*-infected mice compared to the vehicle control. Besides, 25 mg/kg chloroquine significantly (*p* < 0.001) prevented PCV and rectal temperature (Table 3). The prevention of bodyweight reduction was significant at the middle and upper doses of the treatment group (*p* < 0.05 at 200 and *p* < 0.01 at 400 and 600 mg/kg) compared to the curative test's control.

### 3.6. The Effect of the Leaf Latex of *Aloe weloensis* in the Prophylactic Test

The finding showed that the leaf latex at the doses of 200 mg/kg (*p* < 0.05) and 400 and 600 mg/kg (*p* < 0.01) significantly reduced the parasitemia level in the prophylactic test compared to the vehicle control. Parasitemia reduction was dose-dependent, and the percentage of suppression was increased with increasing the doses of the leaf latex of *A. weloensis*. Similarly, all tested doses of *A. weloensis* leaf latex significantly (*p* < 0.01) increased the mean survival time of the mice. The survival time of the mice treated with the latex at 200 mg/kg dose was significantly (*p* < 0.01) lower than the standard drug (Table 4).

## 4. Discussion

The antimalarial activity of the leaf latex of *Aloe weloensis* was evaluated against *Plasmodium* parasites. The in vitro test was evaluated on the chloroquine-sensitive 3D7 strain of the parasite. In contrast, in vivo tests were evaluated on *P. berghei* infected mice since *P*. *berghei* produce diseases similar to human *Plasmodium* infection and sensitivity to standard drug chloroquine [4, 17, 28].

In this study, the leaf latex showed the potent antimalarial activity against the 3D7 strain of *P. falciparum*. Parasite inhibition was dose-dependent, with IC_50_ values of the leaf latex and chloroquine 9.14 and 0.02 *μ*g/mL, respectively. According to a previous study by Satish and Sunita [19], the leaf latex of *A. weloensis* was active (IC_50_ = 5–50 *μ*g/ml) against the 3D7 strain of *P. falciparum*. The parasite growth inhibition calls for further investigation in the curative and prophylactic model against *P. berghei*-infected mice, since in vivo models allow the possible bioactivation and the likelihood of the immune system to eradicate the infection, unlike in vitro studies [4, 6, 27].

Plant extracts are considered active when reduction or percentage suppression in parasitemia is ≥ 30% or significant prolonging the survival time of treated mice compared to the vehicle control [29–31]. Thus, the leaf latex of *A. weloensis* was found to be active against *P. berghei* infected mice.

A curative test was employed in the current study to assess the leaf latex effect in late *Plasmodium* infection. The finding showed that the curative effect of the latex was significant (*p* < 0.001) at all doses compared to the vehicle with % suppression of 36% (200 mg/kg), 58% (400 mg/kg), and 74% (600 mg/kg). This confirmed that the leaf latex of *A. weloensis* endowed efficacy in the late stages of *Plasmodium* infection. The relatively less chemosuppression activity (36%) at 200 mg/kg dose of the leaf latex is possibly due to less accumulative efficacy to bring high chemosuppression. The latex at the 400 mg/kg (58%) and 600 mg/kg (74%) showed greater parasite suppression, implying the latex dose-dependent curative effect. Compared to the previous 4-day suppressive test (*p* < 0.01) [16], the leaf latex of *Aloe weloensis* showed greater curative potential (*p* < 0.001) in the late stage of *Plasmodium* infection in the curative test.

Phytoconstituents present in the latex may block parasite growth and replication. Alkaloids endowed the antimalarial effect by blocking detoxification of heme and protein synthesis in *P. falciparum* [32, 33]. Quinine is an alkaloidal antimalarial drug isolated from *Cinchona* bark. It is useful in treating multidrug-resistant malaria and serving as the lead compound for chloroquine derivatives [34]. Phytosterols and flavonoids showed an outstanding activity against *Plasmodium* parasites by boosting host immunity [35].

In this study, all doses of the latex significantly (*p* < 0.01) improved the mean survival time of the mice compared to the negative control in the curative test. This finding might indicate that the latex suppressed *P. berghei* and reduced the parasite's overall pathologic effect on the mice. The survival time of the mice treated by various doses of the latex longer in the curative test is compared to the previous 4-day suppressive test [16], possibly due to the longest mean survival time of the mice strongly associated with the maximum parasitemia inhibition. According to the previous study by Basir et al., the leaf latex of *A. weloensis* was active as the latex prolonged mean survival time beyond 12 days [36].

In addition, packed cell volume and rectal temperature of mice were used to predict the effectiveness of the test compounds. Contrary to humans, mice's body temperature was decreased while increasing parasitemia due to a decrease in the metabolism of infected mice [6, 36]. In this study, the latex doses at 400 and 600 mg/kg showed a significant (*p* < 0.01) protective effect in rectal temperature of *P. berghei* infected mice. This could probably be due to the latex's preventive effects in some pathological processes that cause a reduction in internal body temperature and augment the immune system and metabolic rate of infected mice.

Packed cell volume reduction is one feature of *P. berghei* infected mice and was determined to evaluate the effectiveness of *Aloe weloensis*. In both humans and mice, escalating parasitemia destroys infected RBCs, clearance of uninfected RBCs, and erythropoietic suppression [37]. Packed cell volume was monitored before infection and on day four after infections to predict the effectiveness of the study plant. The present study showed that medium and high doses of the latex significantly (*p* < 0.01) prevented PCV reduction compared to vehicle control. This effect is in line with the pack cell volume protection effect of the *Aloe megalacantha* [38]. However, the lower dose was devoid of the significant prevention effect of red blood cells hemolysis. This might be due to the low concentration of bioactive molecules at the lower dose relative to the other doses. The prevention of packed cell volume reduction might be due to the leaf latex's antiplasmodial effect against the parasitized RBCs and the causative parasite, thereby sustaining the availability of the new RBCs produced in the bone marrow [39, 40].

The bodyweight loss in the experimental animals is due to the appetite-suppressing effects of the parasite [36]. Similarly, the present finding showed that the latex of *A. weloensis* was significant in preventing *P. berghei*-induced weight loss in mice at all tested doses. The findings of this study showed that packed cell volume, rectal temperature, and bodyweight of infected mice were concordant with the previous 4-day suppressive test [16].

In this study, the result showed significant dose-dependent parasitemia reduction of all doses of the leaf latex of *A. weloensis* in the prophylactic test. Parasitemia suppression was 38% at 200 mg/kg, 46% at 400 mg/kg, and 57% 600 mg/kg doses of the latex. The mean survival time of the mice treated by all doses of the latex was significantly prolonged relative to the control, but the survival time of the mice treated by low dose was significantly lower than the standard drug. The result of this study showed that the leaf latex of the plant might prevent transmission of the *Plasmodium* parasite.

## 5. Conclusion

The findings of the present study confirmed the prominent antimalarial activity of the leaf latex of *Aloe weloensis* against the 3D7 strain of *P. falciparum* and *P. berghei* and corroborate its use in folk medicine. The medium and higher doses of the latex showed a greater prophylactic and curative effect. Therefore, an advanced study is required for organ toxicity study and to identify, characterize, and isolate the bioactive compounds that possess the antimalarial activity.

## Figures and Tables

**Figure 1:** *P. falciparum* growth inhibition effect of the leaf latex of *A. weloensis*.

**Table 1:** Percentage of the free radical scavenging activity of the leaf latex of *Aloe weloensis*.

Concentration (*μ*g/ml)	% of inhibition	
	Ascorbic acid	Leaf latex
12.5	26.03 ± 0.16	9.21 ± 0.37
25	37.82 ± 0.23	21.67 ± 0.71
50	54.56 ± 0.52	33.14 ± 0.53
100	70.21 ± 0.32	47.01 ± 0.41
200	79.38 ± 0.45	68.01 ± 0.31
400	95.13 ± 0.34	83.54 ± 0.27
IC50 (*μ*g/ml)	2.97	10.25

The data are expressed as mean ± standard error of the mean (*n* = 3).

**Table 2:** Parasitemia level, % suppression, and survival time of infected mice treated by the leaf latex of *A. weloensis* in the curative test.

Groups	% parasitemia	% suppression	Survival time (days)
10 ml/kg NC	76.85 ± 0.61	00.00	8.12% ± 0.41
25 mg/kg CQ	00.00 ± 0.00	100.00^a3b3c2d2^	30.00 ± 0.00^a3b2^
200 mg/kg LL	40.37 ± 0.71^a3e2^	36.17^a3e3^	12.72 ± 0.45^a2e2^
400 mg/kg LL	30.25 ± 0.45^a3e2^	57.69^a3e2^	20.14 ± 0.62^a2^
600 mg/kg LL	23.65 ± 0.57^a3e1^	73.51^a3e2^	24.87 ± 0.73^a2^

Data are expressed as mean ± standard error of the mean; *n* = 6. ^a^Compared to vehicle; ^b^compared to 200 mg/kg; ^c^compared to 400 mg/kg; ^d^compared to 600 mg/kg; ^e^compared to 25 mg/kg CQ. ^1^*p* < 0.05, ^2^*p* < 0.01, and ^3^*p* < 0.001 with respect to vehicle control. CQ, chloroquine; LL, leaf latex; NC, negative control.

**Table 3:** Packed cell volume, rectal temperature, and the bodyweight of infected mice treated by the leaf latex of *A. weloensis* in the curative test.

Groups	PCV		Temperature		Bodyweight	
	Day 0	Day 4	Day 0	Day 4	Day 0	Day 4
10 ml/kg NC	49.60 ± 1.36	40.60 ± 1.81	37.12 ± 0.16	29.64 ± 0.36	28.80 ± 0.37	24.760 ± 0.23
25 mg/kg CQ	48.12 ± 0.10	53.20 ± 0.37^a3b1^	35.60 ± 0.73	37.42 ± 0.12^a3^	27.60 ± 0.51	32.60 ± 0.73^a3^
200 mg/kg LL	48.00 ± 0.71	42.00 ± 0.95^c1^	36.58 ± 0.13	32.38 ± 0.31^c1^	27.00 ± 0.71	27.24 ± 0.37^a1^
400 mg/kg LL	48.80 ± 0.73	46.80 ± 0.63^a2^	36.54 ± 0.18	34.36 ± 0.31^a2^	26.80 ± 0.37	29.60 ± 1.52^a2^
600 mg/kg LL	49.00 ± 0.56	47.10 ± 1.08^a2^	36.54 ± 0.18	36.02 ± 0.07^a2^	28.60 ± 0.51	31.80 ± 0.68^a2^

Data are expressed as means ± standard error of the mean; *n* = 6. ^a^Compared to vehicle; ^b^compared to 200 mg/kg; ^c^compared to 25 mg/kg CQ. ^1^*p* < 0.05, ^2^*p* < 0.01, and ^3^*p* < 0.001 with respect to vehicle control. Day 0, weight, temperature, and packed cell volume pretreatment on day zero. Day 4, posttreatment on day five. CQ, chloroquine; LL, leaf latex; NC, negative control; PCV, packed cell volume.

**Table 4:** Parasitemia level, % suppression, and survival time of infected mice treated by the leaf latex of *Aloe weloensis* in the prophylactic test.

Group	% parasitemia	%suppression	Survival time (days)
10 ml/kg NC	65.31 ± 0.17	—	5.72 ± 0.42
25 mg/kg CQ	00.0 ± 00^a3b2^	100	30.45 ± 0.18^a3b2^
200 mg/kg LL	27.42 ± 0.23^a1c1d1e2^	37.87	8.21 ± 0.15^a1d1e2^
400 mg/kg LL	16.52 ± 0.18^a2b1^	46.29	14.10 ± 0.31^a2^
600 mg/kg LL	12.12 ± 0.41^a2b1^	56.68	17.50 ± 0.22^a3b1^

Data are expressed as means ± standard error of the mean; *n* = 6. ^a^Compared to vehicle; ^b^compared to 200 mg/kg; ^c^compared to 400 mg/kg; ^d^compared to 600 mg/kg; ^e^compared to 25 mg/kg CQ. ^1^*p* < 0.05, ^2^*p* < 0.01, and ^3^*p* < 0.001 with respect to vehicle control. CQ, chloroquine; LL, leaf latex; NC, negative control.

## Data Availability

The datasets used/or analyzed to support the findings of this study are available from the corresponding author upon request.

## Abbreviations

CQ: Chloroquine
DPPH: Diphenyl-1-picrylhydrazine
IC50: Inhibitory concentration 50
LD50%: Lethal dose 50
LL: Leaf latex
MST: Mean survival time
NC: Negative control
OECD: Organisation for Economic Co-operation and Development
PCV: Packed cell volume
RBCs: Red blood cells
PRBCs: Parasitized red blood cells
TW80: Tween-80 in distilled water.
